# High-Performance Concrete Strength Prediction Based on Machine Learning

**DOI:** 10.1155/2022/5802217

**Published:** 2022-05-28

**Authors:** Yanning Liu

**Affiliations:** Shanxi Polytechnic College, Taiyuan 030006, China

## Abstract

High-performance concrete is a new high-tech concrete, produced using conventional materials and processes, with all the mechanical properties required for concrete structures, with high durability, high workability, and high volume stability of the concrete. The compressive strength of high-performance concrete has exceeded 200 MPa. 28-d average strength between 100 to 120 MPa of high-performance concrete has been widely used in engineering. Compressive strength is one of the important parameters of concrete, and carrying out concrete compressive strength prediction is of high reference value for concrete design. Eight variables related to concrete strength are used as the input of the machine learning algorithm, and the compressive strength of HPC is used as the object of study. 60 samples are constructed as the dataset by concrete preparation, and the prediction of compressive strength of HPC is carried out by combining the XGBoost algorithm. In addition, SVR algorithm and RF algorithm are also performed on the same dataset. The results show that the XGBoost model has the highest prediction accuracy among the three machine learning models, and the XGBoost algorithm scores 0.9993 for **R**^2^ and 1.372 for RMSE on the test set. The XGBoost algorithm has high prediction accuracy in predicting the compressive strength of HPC, and the choice of model is important for improving the prediction accuracy.

## 1. Introduction

High-performance concrete (HPC) is a new type of high technology concrete, which is produced using conventional materials and processes [1]. The production process requires the incorporation of external admixtures that improve the properties of concrete, adding high durability, workability, and volumetric stability on top of improving the mechanical properties of concrete. The excellent performance of HPC makes it widely used in various fields of the construction industry. A lot of practical experience in engineering proves that controlling the quality of concrete is extremely important for the safety and durability of building structures. As a core element of concrete quality control and an important basis for structural design and construction, the 28-d compressive strength of concrete specimens after curing is a key parameter in the design of concrete structures and an important indicator of the engineering performance of HPC. It is a key parameter in the design of concrete structures and an important indicator of the engineering performance of HPC. In engineering practice, whether the strength of HPC meets the design requirements is the primary issue, the ordinary orthogonal experimental method to determine the compressive strength of HPC is relatively time-consuming, and the procedure is cumbersome and costly. In order to meet the requirements of timely presumption and early control of concrete quality in construction, it is important to develop and improve the early concrete strength prediction technology adapted to the actual project and continuously improve the prediction accuracy to improve the construction quality and speed up the construction schedule. Therefore, it is of high economic value and practical guidance to predict the strength of HPC quickly and accurately [2].

As one of the most widely used and largest construction materials for modern engineering structures in the world today, concrete materials have played an important role in the process of economic development and social progress. With the development of capital construction and the advancement of construction technology, the scale of engineering construction is becoming more ambitious, the structural forms are more replicated, and the requirements of the construction industry for concrete performance have increased. HPC is developed on the basis of high-strength concrete, and the definition of HPC varies from country to country. In general, HPC should have high permeability, high volumetric stability, appropriately high compressive strength, and good workability. It can be seen that the prediction of the strength of HPC not only is of theoretical value, but also has a high practical engineering value.

In recent years, with the rapid development of artificial intelligence technology, various industries are combining new artificial intelligence technologies for self-empowerment, and engineering-based research based on machine learning and deep learning has continued. Many machine learning theories have been applied to concrete-related research, mainly including artificial neural networks [3], support vector [4], and integration algorithms [5]. Erdal et al. [6] predicted the strength of HPC based on wavelet transform neural network model, and the prediction accuracy was good. Yuan et al. [7] proposed two hybrid neural networks, genetic optimization BP neural network, and ANFIS, to predict the strength of concrete, and compared the results with the ordinary BP neural network model, and the results showed that the prediction accuracy of the hybrid neural network model was greatly improved. Daneshvar and Behnood [8] used random forest algorithm to build a dynamic-elastic mode prediction model for asphalt concrete, and the prediction accuracy could reach 94.62%. Ren et al. [9] proposed a convolutional neural network for semantic segmentation of cracks based on computer vision technology, which provides a new method for health monitoring of tunnels. Cui et al. [10] introduced the attention mechanism into the semantic segmentation task of concrete cracks and proposed a convolutional neural network with AttUnet to achieve accurate semantic segmentation of cracks. Chun et al. [11] carried out the study of internal damage of reinforced concrete structures based on random forest algorithm and achieved accurate prediction results. Chou et al. [12] proposed an improved least squares support vector regression algorithm to improve the accuracy of high-performance concrete compressive strength prediction by parameter optimization. Behnood et al. [13] used M5P algorithm to study high-performance concrete compressive strength prediction by constructing model trees from high-latitude data. Zhou et al. [14] used 10 supervised learning algorithms for rock-burst prediction based on 246 sets of rock-burst cases and compared the prediction results of different algorithms.

Concrete-related research based on machine learning has been carried out and achieved some results. Farouk and Jinsong [15] explored machine learning in concrete strength prediction by using four machine learning algorithms, SVM, ANN, MLR, and SWR, to predict the strength of UHPC-NSC interface bond. Kim et al. [16] used CatBoost algorithm to predict FRP-concrete interface bond strength as an improved ensemble machine learning method with better performance metrics when compared with histogram gradient boosting algorithm and extreme gradient boosting algorithm and random forest. Tran et al. [17] used six machine learning models such as GB algorithm, XGB algorithm, support vector regression, and hybrid models with particle swarm optimization, i.e., GB_PSO, XGB_PSO, and SVR_PSO, to predict the strength of recycled compressive strength of concrete. Researchers often compare multiple methods to select the optimal model for concrete strength prediction, but there is a lack of case studies on strength prediction of HPC. In this paper, three machine learning algorithms, RF, SVR, and XGBoost, are used to predict the compressive strength of HPC based on the quality characteristics of HPC. Also, cement dosage, age, water, coarse aggregate, fine aggregate, high-efficiency water reducing agent, fly ash, and mineral powder are used as multiple features and input to construct the machine learning model dataset. Training testing, along with comparing the accuracy of different models in applying to the prediction of compressive strength of HPC, and selecting the optimal model applicable to the prediction of compressive strength of concrete, can also be helpful in constructing the machine learning model dataset.

## 2. Concrete Preparation and Datasets

The concrete specimens were prepared using Southern P-O 42.5 grade cement, Guodian Shuang liao Class I fly ash, Huibei Mining crushed stone with continuous grading from 5 to 31.5 mm, Rong Shun quartz sand with fineness modulus of 2.29, and poly-carboxylic acid high-efficiency water reducing agent from Wuhan Harbor Research Institute Co. The powdered poly-carboxylic acid high-efficiency water reducing agent (water reduction rate of 23%) and alkylphenol ethylene oxide compound air-entraining agent were added during mixing, in which the high-efficiency water reducing agent accounted for 0.2%∼0.8% of the cement mass and the air-entraining agent accounted for 0.8%∼1.2% of the cement mass. The amount of HPC and air-entraining agent and the ratio of sand, cement, and water were adjusted experimentally according to the desired workability, including flowability, cohesiveness and water retention, and slump measured using a slump cone.

The HPC molding and mixing procedure include starting the mixer, putting in cement, fly ash, quartz sand, and other powders, dry mixing three minutes, adding water and water reducing agent, and mixing for three to five minutes. After the mixing is completed, the mix is poured into the steel mold, and after shaking and smoothing, the mold is covered with plastic film to prevent rapid moisture dissipation and left to stand at room temperature for 48 hours before demolding. The slump was measured to be 220 mm, with good fluidity, cohesion, and water retention. The test method was in accordance with GB/T 50081-2016 “test method for mechanical properties of ordinary concrete,” and a total of 60 sets of data samples were produced.

A scientific and reasonable dataset is the key to achieve accurate prediction of concrete strength, which is mainly related to cement. Concrete strength is mainly related to variables such as cement dosage, age, water, coarse aggregate, fine aggregate, high-efficiency water reducing agent, fly ash, and mineral powder. Therefore, the values of the above indicators need to be measured during the preparation of the specimens as the input to the machine learning model, and the output is the compressive strength value of the concrete.

## 3. Predictive Methods of HPCS

### 3.1. RF Algorithm

Bagging is the process of training multiple base classifiers on a dataset and then voting on the results obtained from the base classifiers as the final classification result. Random forest (RF) algorithm is an extended variant of bagging. Due to its excellent performance in data classification, it is often used in recent years for strength prediction of various types of concrete [18]. Based on the integration of the decision tree as the base classifier, RF further introduces random attribute selection in the training process of the decision tree. It selects the splitting feature by measuring the impurity of the feature division result and calculating the information gain. From the root node, according to the feature division condition and the principle of minimum purity of nodes, splitting downward until the rule is satisfied, the final prediction result is the weighted average of the results of each decision tree.

Information entropy is often used as a measure of the purity of a dataset. Let the proportion of the *k*-th class of data to all datasets *X* be *p*_*k*_(*k*=1,2,…, *n*); then, the information entropy of the dataset *X* is defined as equation (1) [19]. The smaller the value of *H*(*X*), the less chaotic and purer the dataset *X*.

(1) $$\begin{array}{c} H\left(X\right)=-\sum_{k=1}^{n}p_{k}\log_{2}p_{k}. \end{array}$$

Assuming that the discrete feature *α* is used to classify the dataset *X*, *I* classification results are generated, where the *I*-th classification result contains all the data, denoted as *X*_*I*_. The information entropy of *X*_*I*_ is calculated according to equation (1), and considering that different classification results contain different amounts of data, each classification result is given a weight of |*X*_*I*_|/|*X*|, indicating that the more data the classification result has, the greater the role of the classification result, so the information gain obtained by using feature *α* to divide the dataset *X* is calculated in equation (2). Generally speaking, the larger the value of Gain(*D*, *α*) is, the more the complexity of the dataset is reduced after the feature a is used for splitting, and the more obvious the classification result is.

(2) $$\begin{array}{c} \text{Gain}\left(D,\alpha \right)=H\left(X\right)-\sum_{i=1}^{I}\frac{\left|X_{I}\right|}{\left|X\right|}H\left(X_{I}\right). \end{array}$$

RF randomly selects *m* subsamples from the original dataset with put-back, and then randomly selects *k* features when training a single decision tree, and chooses the optimal features from these *k* features to split the nodes, which makes the random forest model not easily overlearn the features of the training set and reduces the variance of the model.

### 3.2. SVR Algorithm

The support vector regression algorithm is an application of SVM (support vector machine) to the regression problem, where the SVR creates a “spacing band” on both sides of the linear function with *ε*, also called the SVR creating a “spacing band” on both sides of the linear function with a spacing of *ε*, also known as tolerance bias, and does not calculate losses for all samples falling into the spacing band; i.e., only the support vector affects its functional model, and the optimized model is derived by minimizing the total losses and maximizing the spacing [20]. The basis consists of two main principles. One is that the model allows *ε* error between the predicted value *f*(*x*) and the true value *y*. The second is that the loss function of the model is parameter updated only when the absolute value of the difference between *f*(*x*) and *y* is greater than varepsilon. The SVR model constructs a band of model parameter nonupdating regions with *f*(*x*) as the center and ±*ε* as the broadband.

Given the training data *D*={(*x*_1_, *y*_1_), (*x*_2_, *y*_2_),…, (*x*_*m*_, *y*_*m*_)}, the regression model *f*(*x*)=*w*^*T*^*x*+*b* is obtained by machine learning so that *f*(*x*) is as close to *y* as possible. For the sample (*x*, *y*), traditional regression models usually calculate the loss directly based on the difference between the model output *f*(*x*) and the true output *y*. The loss is 0 when and only when *f*(*x*) is exactly equal to *y*. It follows that the SVR problem can be described by

(3) $$\begin{array}{c} L\left(w,y_{i},f\left(x_{i}\right)\right)=\underset{w,b}{\min}\frac{1}{2}w^{2}+C\sum_{i=1}^{m}l\left(f\left(x_{i}\right)-y_{i}\right), \end{array}$$

where *w* is the normal vector, *C* is the regularization constant, *L* is the model optimization objective function, *f*(*x*_*i*_) is the predicted value of the model, and *y*_*i*_ is the true label value of the data.

The SVR algorithm uses a kernel function that allows mapping to a higher dimensional space and thus solves the classification of nonlinearities. The classification idea is simple, which is to maximize the interval between the sample and the decision surface. In addition, the SVR algorithm has better classification results. However, it is more difficult for processing large samples for large-scale data training, while the concrete strength prediction problem studied in this paper does not belong to large-scale data training and can achieve better prediction results using SVR algorithm.

### 3.3. XGBoost Algorithm

The idea of boosting algorithm is to integrate many weak classifiers together to form a strong classifier. XGBoost is also known as extreme gradient boosting. It is widely used in classification and regression fields because of its fast, efficient, and accurate operations and strong generalization ability [21]. Parameters such as the amount of cement used in concrete can affect its strength and durability, and XGBoost is often used to study the complex interrelationships between multiple influencing factors and their performance indicators [22]. XGBoost supports user-defined objective functions and evaluation functions, and for samples with missing values of features, it can automatically learn its splitting direction. The core concept is to learn new features by adding trees, fitting the residuals of the final prediction, and then obtaining the sample scores, which can be summed up for each tree to obtain the final prediction score of the sample. For *n* labeled samples with *m* features, it uses *G* additive functions to predict scores, and the specific process is shown in

(4) $$\begin{array}{c} y_{\text{pre}}=\sum_{g=1}^{G}f_{g}\left(x_{i}\right),\;f_{g}\in F;\\ F=\left\{f\left(x\right)=w_{q\left(x\right)}\left(q:R^{m}⟶T,w\in R^{T}\right)\right\}, \end{array}$$

where *F* represents the space of regression trees, *f*(*x*) is one of the regression trees, and *w*_*q*(*x*)_ represents the independent structure score of each T-leaf tree. The objective function of XGBoost is defined as

(5) $$\begin{array}{c} L=\sum_{i=1}^{n}l\left(y_{i}^{*},y_{i}\right)+\sum_{g=1}^{G}\Omega \left(f_{g}\right);\\ \Omega \left(f_{g}\right)=\gamma T+\frac{1}{2}\mu w^{2}, \end{array}$$

where *l* denotes the loss function of the model, *Ω* is the regularization term, *T* denotes the number of leaf nodes, *w* is the fraction of leaf nodes, while *γ* and *μ* represent the control coefficients to prevent overfitting. To speed up the optimization, a Taylor second-order expansion can be used, as shown in

(6) $$\begin{array}{c} L\left(t\right)=\sum_{i=1}^{n}\left[l\left(y_{i},y_{i}^{*\left(t-1\right)}\right)+k_{i}f_{t}\left(x_{i}\right)+\frac{1}{2}h_{i}f_{t}^{2}\left(x_{i}\right)\right]+\gamma T+\frac{1}{2}\mu \sum_{i=1}^{T}w_{i}^{2}. \end{array}$$

By adding the loss function of the samples, the samples an be recombined. And finally using the vertex formula to find the optimal *w* and the objective function formula *L* as shown in equation.

(7) $$\begin{array}{c} w_{i}^{\prime }=-\frac{K_{i}}{H_{i}+\mu }\;;\\ L=-\frac{1}{2}\sum_{i=1}^{T}\frac{K_{i}^{2}}{H_{i}+\mu }+\gamma T, \end{array}$$

where *K*_*i*_=∑_*i*∈*I*_*j*__*k*_*i*_ and *H*_*i*_=∑_*i*∈*I*_*j*__*h*_*i*_. XGBoost combines the traditional greedy algorithm with an approximation algorithm to find the best splitting point by enumerating several possible candidates based on the percentile method and then calculating the best splitting point according to equation (7). XGBoost uses various methods to avoid overfitting, such as introducing regularization, row sampling, and feature sampling, and also adds handling of sparse data. In addition, XGBoost has other advantages, such as the ability to perform parallel processing, which results in a significant speedup; a high degree of flexibility, with customizable optimization goals and evaluation criteria; and built-in cross-validation, which allows cross-validation to be used in each boosting iteration. Combining the above advantages of XGBoost in classification algorithms, this paper selects XGBoost as one of the main alternative models for HPCS. The modeling steps of XGBoost are shown in Figure 1.

Firstly, we define the algorithm function and call the XGBoost function to build the network model; then, we set the initial parameters and input the training set to train the model, adjusting the weights every time until the training error is minimized or the required maximum training times are reached; after training, we store the current network file and input the validation set to compare the evaluation metrics to determine whether it is optimal or not, and so on until all parameters are optimal; then, we enter the testing phase and evaluate the model to obtain the corresponding metrics to complete the classification experiment of HPCS.

## 4. Experimental Results and Analysis

For the purpose of selecting the most suitable prediction model for HPCS, this paper uses the comparative experimental method. Specific concrete samples are prepared in the laboratory, and the data are preprocessed after understanding the characteristics of each data, so as to select the model with the best prediction performance based on machine learning theory. The overall technical route is shown in Figure 2.

In order to compare and analyze the performance of three machine learning methods, RF, SVR, and XGBoost, on the concrete compressive strength dataset, this paper selects *R*^2^ and RMSE from the commonly used machine learning evaluation metrics. Where the root mean square error (RMSE) mainly measures the accuracy of the model, the smaller its value, the higher the prediction accuracy of the model. The correlation coefficient (*R*^2^) characterizes the closeness between the predicted value of the model and the true value of the data, and the closer the *R*^2^ is to 1, the higher the prediction accuracy of the model. The mathematical formula is shown in

(8) $$\begin{array}{c} R^{2}=\frac{\sum_{i}{\left(y_{\text{obs}}-y_{\text{pre}}\right)}^{2}}{\sum_{i}{\left(y_{\text{obs}}-\bar{y_{\text{obs}}}\right)}^{2}};\\ \text{RMSE}=\sqrt{\frac{\sum_{i}{\left(y_{\text{obs}}-y_{\text{pre}}\right)}^{2}}{n}}. \end{array}$$

### 4.1. Comparative Analysis of Model Results

Before comparing the prediction results of each model, the *GridSearch* method is used to optimize the parameters of various models for making the prediction results of each model more accurate. The results of the parameter optimization are shown in Table 1. Eight influencing factors such as cement use, age, water, coarse aggregate, fine aggregate, high-efficiency water reducer, fly ash, and mineral powder are selected as input variables, and 28-d compressive strength was taken as the prediction target to construct the initial index system of the high-performance concrete compressive strength prediction model. The original dataset was randomly divided into 10 parts according to the ratio of 8 : 2, of which 80% was used as the training set and the rest as the test set. In this paper, there are 60 sets of data samples, 48 sets are divided into training set, and the remaining 12 sets are test sets. We perform statistical analysis on the prediction results of each model, and the comparison results in test sets are listed in Figure 3.

Analysis of Figure 3 shows that, overall, for the error measure RMSE, the XGBoost model has the lowest error prediction 1.372, followed by RF 2.347 and finally SVR 2.656. In terms of the correlation coefficient *R*^2^, all three models get the desired value; that is, the concrete strength data in this paper are convincing. The correlation coefficient of the XGBoost model reaches 0.9993, reaching the maximum value of the three. The results of these two evaluation indexes fully illustrate the superiority of XGBoost algorithm in HPCS prediction, which can be used as a favorable reference for future prediction work.

### 4.2. Prediction Result Analysis of XGBoost

XGBoost implements a general tree boosting algorithm. In view of the good performance of XGBoost algorithm in HPCS prediction, this paper analyzes the operation results of XGBoost in detail to better illustrate the adaptability of this method.

The statistical results of the comparison between the HPCS prediction results of the XGBoost model and the actual compressive strength are shown in Figures 4 and 5.

When training is performed, the XGBoost algorithm achieves good results, and the actual values are almost indistinguishable from the predicted values. Therefore, in order to visualize the prediction effect of the training set, Figure 4 shows the actual values as the horizontal coordinates and the predicted values as the vertical coordinates, and the distribution of each data point basically coincides with the line *y*=*x*. The composition of concrete strength data in the training set ranges from 20 MPa to 70 MPa, the RMSE is 0.341, and *R*^2^ is 0.9989 after XGBoost training. This indicates that XGBoost has a very excellent prediction performance in the training phase.

Figure 5 reveals that although XGBoost achieves good outcomes on the training set, there is no overfitting, and the performance on the training set is also outstanding. In general, for different strengths of high-performance concrete, the predictions of the XGBoost model are very close to the true values of the test set, and the dashed and solid lines are generally in the same direction. The RMSE on the training set is 1.372, while the *R*^2^ is 0.993. The trend of the two lines in the figure shows that the strength prediction performance of concrete with strengths in the interval of 40–50 MPa is better than that of 50–70 MPa. Judging from the performance on the training set and validation set, the XGBoost prediction model has strong adaptability and superiority in HPCS prediction and can better guide the prediction of compressive strength of HPC.

The construction industry is pursuing higher and higher quality of construction, and the strength of concrete is often a key influencing factor of that. How to prepare high-performance concrete is an important topic in civil engineering materials science, and a high-performance concrete strength prediction model will greatly dominate the preparation of concrete. As a simple example, with the prediction model, it is possible to filter the dosage range of important indicators such as cement dosage according to the actual demand. This greatly reduces the number of pre-experiments conducted and the time to conduct them, which also saves experimental materials and speeds up the efficiency of experiments. Nowadays, there are still some problems in concrete prediction, such as lack of sample data, lack of representativeness, inability to reflect the sensitivity of input parameters, and narrow scope of application of the model. Concrete prediction, as a typical multivariate, nonlinear system, requires the incorporation of reasonable data processing methods such as machine learning to be performed. This paper uses comparisons to select a better quality method that can better serve HPC in practical engineering for problems such as proportioning optimization.

## 5. Conclusion

With the large-scale development of transportation infrastructure, how to use the available data to make accurate prediction of concrete strength, so as to feed back to optimize the concrete mix design, has become a hot topic of research in the academic and engineering circles nowadays. The strengths of the HPCs we prepared ranged from 20 MPa to 70 MPa. To better investigate the nonlinear relationship between HPCS and the eight influencing factors, machine learning approaches are used to solve this problem. In order to find the most suitable algorithm to strength prediction, three commonly used and effective methods, RF, SVR, and XGBoost, are selected using comparative analysis. Through data preprocessing and parameter optimization, all three methods achieve a nice prediction state, and the results of the study can provide some reference for machine learning in the field of concrete strength prediction research. The *R*^2^ values of the three methods are all above 0.9, and the model fitting effect is good. By comparing the performance capability of RF, SVR, and XGBoost algorithms on the same dataset, it is found that XGBoost has the highest prediction accuracy and the lowest RMSE value of 1.372, which can be applied to HPCS prediction.

The prediction method in this paper has high precision; therefore, it will serve the experimental design of the laboratory. In addition, machine learning algorithms can also identify the most sensitive intensity influencers, which can also be used for future research.

## Figures and Tables

**Figure 1:** XGBoost modeling steps.

**Figure 2:** Technical route of HPCS prediction.

**Figure 3:** Comparison of test set evaluation results.

**Figure 4:** XGBoost training set result.

**Figure 5:** XGBoost testing set result.

**Table 1:** Parameter configuration.

Algorithm	Parameter optimization
RF	*n*_estimators = 500, max_depth = 18, min_samples_split = 4
SVR	Kernel = “rbf,” *C* = 1010, gamma = 0.56
XGBoost	*n*_estimators = 500, max_depth = 6, learning_rate = 0.01

## Data Availability

The labeled datasets used to support the findings of this study are available from the corresponding author upon request.
